The article "A Comprehensive Review of Recent Deep Learning Techniques for Human Activity Recognition" was published in 2022. Journal: Comput Intell Neurosci.

# A Comprehensive Review of Recent Deep Learning Techniques for Human Activity Recognition

**DOI:** 10.1155/2022/8323962

**Published:** 2022-04-20

**Authors:** Viet-Tuan Le, Kiet Tran-Trung, Vinh Truong Hoang

**Affiliations:** Ho Chi Minh City Open University, 35-37 Ho Hao Hon Street, Ward Co Giang, District 1, Ho Chi Minh City, Vietnam

## Abstract

Human action recognition is an important field in computer vision that has attracted remarkable attention from researchers. This survey aims to provide a comprehensive overview of recent human action recognition approaches based on deep learning using RGB video data. Our work divides recent deep learning-based methods into five different categories to provide a comprehensive overview for researchers who are interested in this field of computer vision. Moreover, a pure-transformer architecture (convolution-free) has outperformed its convolutional counterparts in many fields of computer vision recently. Our work also provides recent convolution-free-based methods which replaced convolution networks with the transformer networks that achieved state-of-the-art results on many human action recognition datasets. Firstly, we discuss proposed methods based on a 2D convolutional neural network. Then, methods based on a recurrent neural network which is used to capture motion information are discussed. 3D convolutional neural network-based methods are used in many recent approaches to capture both spatial and temporal information in videos. However, with long action videos, multistream approaches with different streams to encode different features are reviewed. We also compare the performance of recently proposed methods on four popular benchmark datasets. We review 26 benchmark datasets for human action recognition. Some potential research directions are discussed to conclude this survey.

## 1. Introduction

Human action recognition is one of the most crucial tasks in video understanding. This field has a wide range of applications, such as video retrieval, entertainment, human-computer interaction, behavior analysis, security, video surveillance, and home monitoring. In detail, we want to find handshake events in a movie or offside decisions in a football match and the results are returned automatically. The goal of human action recognition is to recognize automatically the nature of an action from unknown video sequences.

There are some challenges in human action recognition. The view invariance is one of the reasons that make human action recognition more complex. There are some simple datasets having a fixed viewpoint [1, 2] while most of the recent datasets have many viewpoints. In addition, each person has their size and shape as well as posture. They can appear with various clothes and accessories. An action which is performed in an indoor environment with a uniform or static background is easy to recognize than an action that is recorded in a cluttered or dynamic background. In addition, lighting conditions or viewpoints contribute to increase or decrease of the accuracy of recognition. The next problem is intraclass and interclass variations. A human action recognition method must be able to generalize an action over variations within a class and distinguish between actions of different classes. For examples, people have different speeds when they run or walk. The occlusion problem is a hard issue in action recognition because some body parts of humans are disappeared temporarily. For example, some body parts cover other parts or a subject, or a person is hidden behind another person. Temporal variations are also an important challenge because actions are happening for a long time.

Deep learning methods have achieved state-of-the-art results on various problems of computer vision, especially human action recognition. Convolutional neural networks (CNNs) [3] are the neural network that uses convolutional operator in their layers. Convolutional network is used for computing a grid of values such as images while recurrent neural networks (RNNs) [4] are a type of neural network for processing sequential data, such as text and video. In this survey, we focus on proposed methods for human action recognition using deep learning techniques.

### 1.1. Review of Related Survey Articles

Since human action recognition is an attractive problem, many surveys have been done over the last few years. The most popular survey of human action recognition is the work in [5]. Firstly, the authors discussed the local representation and global representation-based methods. Then, three types of action classification approaches were discussed, including direct classification, temporal state-space models, and action detection. However, this study have been conducted over ten years ago, and this survey reviewed methods using handcrafted features.

Zhang et al. [6] provided an overview of human action recognition, interaction recognition, and human action detection methods. The whole part of the survey discussed human action feature representation methods. First, the authors discussed handcrafted action features for RGB, depth, and skeleton data. Then, they reviewed some deep learning-based methods. However, they focused on two-stream networks and long short-term memory methods.

A review of Singh and Vishwakarma [7] focused on human action datasets in the past two decades. They classified these datasets into two classes, namely RGB (Red-Green-Blue) and RGB-D (depth) datasets. They discussed 26 RGB and 22 RGB-D datasets. Two categories of existing methods (handcrafted and learned feature representations) were discussed; however, the main contribution of this work is dataset analysis.

RGB-D data plays a vital role in human action recognition because this data provide color, depth and skeleton data. The performance of human action recognition systems is improved significantly when they exploit depth and skeleton data. With a special focus on RGB-D data, Liu et al. [8] reviewed human action recognition and human interaction recognition based on hand-crafted features. Then, their survey discussed human activity recognition based on deep learning in the next part.

Zhu et al. [9] reviewed over 200 papers about human action recognition. Their survey focused on three different approaches for human action recognition. Firstly, two-stream networks were reviewed. The two-stream methods tried to exploit the temporal relationship between frames because motion information plays a vital role in human action recognition in video. The first stream encodes the spatial information and the second one encodes the optical flow. In this review, the authors focused on recurrent neural networks which were used as a part of a two-stream network while our work discusses RNNs-based methods for human action recognition. Next, 3D CNN-based methods were discussed. 3D CNNs exploit both spatial and temporal information by using a 3D tensor with two spatial and one temporal dimension. The two-stream networks require huge resources to compute, and the 3D CNNs are hard to train. Therefore, they reviewed efficient video modeling which try to reduce computational intensity.

Beddiar et al. [11] reported a survey which discussed human activity recognition approaches in the last ten years. The authors classified human activity recognition approaches into various categories. The first category is the feature extraction process. Both hand-crafted features and feature learning were discussed. Then, they discussed three stages of human activity recognition approaches, including detection, tracking, and recognition. Next, unimodel and multimodel approaches were surveyed. They classify human activity recognition methods into three classes of learning supervision, namely supervised, unsupervised, and semisupervised methods. The review also provided different types of activities. However, the recent deep learning techniques for human activities recognition were not highlighted clearly.

In order to review many different challenges, Jegham et al. [10] reviewed methods which aimed to solve these challenges in human action recognition. Many challenges were discussed such as anthropometric variation, multiview variation, cluttered and dynamic background, interclass similarity, intraclass variability, low-quality videos, occlusion, illumination variation, shadow and scale variation, camera motion, and poor weather conditions. In the second part, the authors reviewed recent action classification methods and popular datasets. They focused on three types of methods, including template-based methods, generative model-based methods, and discriminative model-based methods.

A different survey [12] discussed human pose estimation and the role of it in human action recognition application. Firstly, the survey discussed various types of human pose estimation such as single person, multiperson, 3D human pose estimation, and human pose estimation in videos and depth images. In the remained part, they discussed human pose estimation for action recognition.

A review of single vision and multivision modalities was provided by Majumder and Kehtarnavaz [13]. In the single vision modality section, the authors discussed the approaches which used video data for action recognition. In the next section, the methods using RGB + Depth data were reviewed in multivision modality section. In each modality, both conventional and deep learning approaches were reviewed.

Table 1 provides a summary of recent related surveys. Moreover, some main contributions of this work are discussed.

### 1.2. Contributions of This Survey Article

Human action recognition has a wide range of applications; therefore, many approaches have been proposed using deep learning techniques. We aim to provide a comprehensive survey of recent deep learning techniques for human action recognition. In summary, our main contributions are listed here:

- We discuss the most recent deep learning techniques for human action recognition.
- We provide the first review of convolution-free approaches in the human action recognition field.
- We survey the most popular benchmark datasets for human action recognition
- We provide a comprehensive analysis of proposed methods.

### 1.3. Roadmap of the Survey

As in Figure 1, the rest of the survey is organized as follows. In Section 2, we discuss the most recent deep learning techniques for anomaly detection. Then, we provide two accuracy comparisons of some popular datasets in Section 3.  Section 4 reviews many popular benchmark datasets in the human action recognition field. Finally, we discuss some open research problems and give the conclusion of this survey.

## 2. Recent Deep Learning-Based Methods in Human Action Recognition

In this section, we review recent deep learning-based methods for human action recognition. With the development of large-scale datasets and deep learning, this leads a remarkable growth of models based on deep learning for human action recognition. There are four trends and a new trend has attracted some researchers recently. The first trend is 2D Networks which uses 2D convolutional neural networks in their models, such as TSM [14], TRN [15], and GSM [16]. The second trend is action recognition based on RNN, such as in [17–19]. The third trend is 3D Single Stream Network which uses 3D convolutional kernels in the networks, such as CSN [20] and TSN [21, 22]. The fourth trend is 3D Two-Stream Network which includes a spatial and a temporal stream to encode both structure and optical flow information, such as in [23–26]. Finally, convolution-free approaches based on attention mechanism are a new trend in human action recognition with efficient computation and performance, such as in [27–29] and TimeSformer [30].

### 2.1. Methods Based on 2D CNN

In this part, we will discuss the proposed methods that are based on 2D CNNs. One of the advantages of 2D CNNs is that the computation is cheap [14]. However, 2D CNNs often cannot exploit well the temporal information. Therefore, many approaches try to capture both spatial and temporal information [16, 31, 32]. Optical flow information plays a vital role in action recognition, but the computation cost is expensive. Therefore, in [33–35], the authors tried to compute optical flow with low cost and efficiency.

Two-stream networks are often trained individually with high computational cost. Jiang et al. [31] proposed an efficient method to exploit both spatiotemporal and motion features in a 2D framework, namely STM block. The STM block includes a channel-wise spatiotemporal module (CSTM) and a channel-wise motion module (CMN). The CSTM is used to extract spatiotemporal information. The input feature map *F* ∈ *ℝ*^*N*×*T*×*C*×*H*×*W*^ is reshaped into *F*^*∗*^ ∈ *ℝ*^*NHW*×*C*×*T*^. Then, a channel-wise 1D convolution is applied on input feature maps. A 3D convolutional network can encode local spatial and temporal features. However, they cannot encode ordered temporal information of all clips. A channel-independent directional convolution (CIDC) [32] was introduced to solve this issue. Given input feature map with C channels, CIDC convolve each channel of input feature map with *T*′ filter. The output feature map including spatial and temporal information is obtained by concatenating *C* × *T*′ feature map. Another strategy in action recognition is frame selection. Gowda et al. [36] proposed a smart frame selection method that improved over many state-of-the-art models. The method includes two branches. The first computes a score *δ*_*i*_ for each frame, and the second computes a score *γ*_*i*_ of a pair of frames. Given *n* frames, top *m* frames are chosen using a final score which is multiplied both score *δ*_*i*_ and *γ*_*i*_. Finally, a classifier is used for the final prediction. The authors used the Something-Something-V2 dataset [37] for ablation study. They also experienced on Kinetics [38], UCF101 [39], and HMDB51 [40].

According to the observation, movement variations at motion boundaries are very important in human action recognition. Zhang et al. proposed persistence of appearance (PA) [33] to obtain a map that encodes small motion variations at boundaries. The difference between the optical flow and PA is that PA captures the motion variation without encoding the direction of the movement. Given two frames, eight 7 × 7 convolutions are applied to obtain low-level feature maps *F*_1_, *F*_2_. The *i*-th PA component is computed as *PA*_*i*_(*p*, Δ*t*)=*F*_*i*_(*p*, *t*+Δ*t*) − *F*_*i*_(*p*, *t*), where *F*_*i*_ is the *i*-th feature map. All *PA*_*i*_ are aggregated to a channel *PA*. The PA maps the appearance to the dynamic motion because it maps from three-dimensional to two-dimensional tensor. To exploit motion information, Piergiovanni and Ryoo [34] proposed a convolutional layer to capture the flow of any channel for action recognition without computing optical flow. The proposed fully differentiable convolutional layer has learned parameters that enhance the performance of action recognition systems. Optical flow is an expensive method. Xu et al. [35] proposed a fast network to improve the extraction of optical flow. The optical flow is generated by MotionNet [41] which is an end-to-end trainable network. Moreover, OFF [42] is added to the network to get better optical flow features. The optical flow is computed directly from RGB frames without precalculation or storage. Therefore, both spatial and temporal information are learned by one network.

One of the most popular modules in human action recognition is temporal shift module (TSM) [14]. TSM has the complexity of a 2D CNN but obtains the performance of 3D CNN. In addition, this module can insert into a 2D CNN without extracomputation and parameters. Given a tensor with *C* channels and *T* frames. A part of the channels is shifted by −1, and another part is shifted by +1. The rest of the tensor is unshifted. The TSM can be inserted before convolutional layer or residual block, but the spatial features may be harmed because the information is lost. To deal with this problem, the TSM is inserted into a residual branch in a residual block. To exploit the temporal relations between frames in video, Zhou et al. [15] proposed a temporal relation network (TRN) which predict human-object interactions in the Something-Something dataset accurately. Their paper show that the TRN outperformed two-stream network as well as 3D convolution networks. The pairwise temporal relation is computed as *T*_2_(**V**)=*h*_*ϕ*_(∑_*i*<*j*_*g*_*θ*_(*f*_*i*_, *f*_*j*_)), where **V**={*f*_1_, *f*_2_,…, *f*_*n*_} is the video with *n* frames. The functions *h*_*ϕ*_ and *g*_*θ*_ is used to fuse the frame features. Moreover, The function captured frames relations at different scale is described as *MT*_*N*_(*V*)=*T*_2_(*V*)+*T*_3_(*V*)+⋯+*T*_*N*_(*V*), where *T*_*d*_ is temporal relationship of *d* frames. A 2D convolution neural network (CNN) has smaller parameters and fast computation than a 3D CNN. However, a 2D CNN usually captures spatial information. Sudhakaran et al. proposed a gate shift module (GSM) [16] which is an 2D CNN to capture spatial and temporal features. The input is applied a spatial convolution. Then, a grouped spatial gating is computed. The 2D convolution ouput is split into group-gated features and residual. The gated features are group-shifted and fused with the residual. The spatial and temporal information is exploited by a learning spatial gating.

In a different approach to abovementioned methods, Zhang et al. [43] applied video super-resolution to human action recognition by introducing two video super-resolution (SR) modules, namely spatial-oriented SR (SoSR) and temporal-oriented SR (ToSR). The low-resolution input video is enhanced by two proposed modules. The input of the recognition network includes the output of the SoSR and the optical flow computed from the output of the ToSR module.

### 2.2. Methods Based on RNN

CNNs are popular models for image representation. They are also used to learn action representation in videos [14–16]. However, they often work well with short videos [33, 34], since only spatial features are captured and motion information of action are not encoded. To encode longer motion in video, some approaches have used RNNs, and long-short term memory (LSTM), such as in [17–19]. RNN is widely used in sequence data like video, and text. LSTM is a special version of RNN with the capability of learning long-term information. In addition, LSTM is combined with an attention mechanism [44] or is used in a three-stream network [45, 46] for action recognition.

With video data, RNNs and LSTM requires high memory storage and computation cost. A compact LSTM model (TR-LSTM) [17] was proposed to solve this issue. The TR-LSTM use the tensor ring decomposition to reconstruct the input-to-hidden layer of the recurrent network. In the tensor ring decomposition, the first and last tensors are connected circularly and constructed in a ring-like structure. A densely-connected bi-directional LSTM (DB-LSTM) network [18] is used to represent the spatial and temporal information of human actions. The goal of DB-LSTM is to capture the spatial, short-term, and long-term patterns. The spatial and short-term patterns are extracted by a sample representation learner module, and the long-term patterns are exploited by a sampling stack. Another work, named correlational convolutional LSTM (*C*^2^ LSTM) [19] aims to exploit both spatial and temporal information of human action video. The basic spatial features are extracted by two parallel convolutional networks, and then, these features are used as input for the *C*^2^ LSTM module. The *C*^2^ LSTM extracts the spatial and temporal information as well as the time relation by using cross-correlation inside the LSTM.

A three streams network was proposed by Liu et al. [45] for human action recognition. The network includes a spatial stream, a temporal stream, and a spatial-temporal saliency stream. These streams are used to extract appearance information of RGB frames, motion information of optical flow frames, and spatiotemporal foreground information of objects from spatiotemporal saliency maps. In addition, they proposed three attention-aware LSTMs to exploit the relationship between frames. Another three-stream network [46] processes different frame rates for human activity recognition. The first stream operates at a single frame rate and the second stream processes at low frame rates. Both streams are used to capture spatial features. The third stream processes at high frame rates to capture temporal features. The output of the previous step is fed into two LSTM layers. This makes the proposed model deeper. Instead of using the LSTM layer, the authors use an attention mechanism to capture temporal information.

To extract the salient features of human action videos, Ge et al. [44] introduces an attention mechanism and convolutional LSTM. A convolutional network is used to extract features of the input video. Then, a combination of LSTM and a spatial transformer network extracts salient features. The final classification is obtained by a convolutional LSTM. The proposed combination can select salient localities effectively while getting higher accuracy than soft attention and using less calculation than hard attention.

### 2.3. Methods Based on 3D Single-Stream Network

In this part, we will discuss 3D convolution-based models. These methods obtain good results since 3D CNN extracts spatial and temporal information from action video directly.  Figure 2 is an example of single-stream network architecture. The input frames are fed into a 3D single-stream network to extract both spatial and temporal features.

Tran et al. [20] proposed a channel separated convolutional network (CSN) which employs 3D group convolution. The CSN is defined as 3D CNNs; however, only 1 × 1 × 1 conventional convolutions or *k* × *k* × *k* depthwise convolutions are used. In detail, the conventional convolutions are used for channel interaction and depthwise convolutions are used for local spatiotemporal interactions. In their work, a 3 × 3 × 3 convolution from the bottleneck block by a pair of a 1 × 1 × 1 convolution and a 3 × 3 × 3 depthwise convolution to get a interaction-preserved channel-separated bottleneck block. Moreover, the 1 × 1 × 1 convolution in the previous pair convolutions is removed to obtain interaction-reduced channel-separated bottleneck block. The authors also applied group convolution to ResNet blocks. Two 3 × 3 × 3 convolutional layers of simple ResNet block are replaced by two 3 × 3 × 3 grouped convolutions or a set of one 1 × 1 × 1 convolution and two depthwise convolutions. 3D convolutional neural networks have high training complexity and huge memory cost. In order to resolve this problem, Zhou et al. [47] proposed a combination of 2D and 3D convolution, namely mixed convolutional tube (MiCT). The deep MiCT is an end-to-end network which receives RGB video sequences as inputs. The whole network includes four MiCTs and a global pooling in the last layer of the network. This pooling allows the network to accept any length videos as inputs. Each MiCT block receives an 3D signal. The input process by a 3D convolution to extract spatial-temporal feature maps. The extracted features are passed through a 2D convolution to compute the final feature maps. The MiCT-Net uses fewer 3D convolution, but it obtains deeper feature maps. Instead of combining 2D and 3D convolution, a new spatiotemporal architecture fused 2D and 3D architectures to improve spatiotemporal representation. Diba et al. proposed holistic appearance and temporal network (HATNet) [48] which exploits semantic information at different levels. HATNet uses 2D convolutional blocks to encode the appearance information of individual frames in a video clip. In addition, the 3D convolutions extract temporal information in a batch of frames. ResNet18 and ResNet50 was used in HATNet for 3D and 2D modules, respectively. The output feature maps of each 2D and 3D block are merged; then, a 1 × 1 × 1 convolution is applied to reduce the channel of features. With prestraining on HVU dataset [48], the HATNet obtained 97.8% and 76.5% on UCF101 [39] and HMDB51 datasets [40], respectively.

The video usually has repeating information, and the temporal squeeze network [21] can map the movement information from a long video into a set of few frames. Given a video *X* with K frames, a frame-wize *z* is obtained by applying the squeeze operation. The output of squeeze operation is fed into a excitation operation. Global average pooling is used to implement the squeeze operation while the excitation operation is implement by two fully connected layers and two activation functions. The shorter sequence frames *Y*′ is obtained by projecting the flattened vector of *X* onto the hyperplane **A**, where **A** is computed from the output of the excitation operation. To reduce the computational cost of motion feature, a FASTER-GRU network [49] aggregates the temporal information. The FASTER framework uses an expensive model and a lightweight model to exploit the information of the action and scene, respectively. The FAST-GRU aims to learn the features from multiple models. This network maintains the resolution of feature maps to exploit more spatial-temporal information. A fully connected layer is replaced by a 3D 1 × 1 × 1 convolution. The proposed method was evaluated on Kinetics [38], UCF101 [39], and HMDB51 datasets [40]. A combination of 3D convolution neural network and long-short term memory [50] is used to capture low-level spatial-temporal feature and high level temporal feature. The proposed network used Inception 3D CNN [38] to extract spatial features and low-level motion features from a sequence of frames. Then, the output of the I3D model is fed into a LSTM network to exploit high-level spatial features. Temporal information plays a vital role in human action recognition; however, this information still has challenging problems. A temporal difference network (TDN) [51] was proposed to capture multiscale temporal information. In addition, TDN in an end-to-end model that captures both short-term and long-term motion information. Given *T* frames *I*=[*I*_1_,…, *I*_*T*_], a 2D CNN is used to extract features *F*=[*F*_1_,…, *F*_*T*_]. A short-term and long-term TDM is applied to exploit short-term and long-term motion. To capture the short-term motion, a stacked RGB difference of frame *I*_*i*_ is downsampled using an average pooling, then extracted motion information with a 2D network. The feature is upsampled to match the size of RGB features. In the long-term TDM, the aligned temporal difference is computed, and then fed into a multiscale module to extract long-range motion information. Features are enhanced by a bidirectional cross-segment temporal difference. The TDN framework with ResNet backbone [52] was evaluated on Kinetics-400 [38] and Something-Something-V1-V2 [37]. Instead of computing the optical flow frame-by-frame, the proposed MotionSqueeze module [53] learned motion features by a light-weight learning technique. The module contains three parts, namely correlation computation, displacement estimation, and feature transformation. The correlation score is defined as *s*(*x*, *p*, *t*)=*F*_*x*_^(*t*)^ · *F*_*x*+*p*_^(*t*+1)^, where *F*^(*t*)^ and *F*^(*t*+1)^ are two input feature maps. Then, motion information is estimated in the displacement estimation module and a confidence map of correlation is obtained from the correlation. The concatenation of displacement map and the confidence map is used as the input of the feature transformation. The feature transformation converts the input into an effective motion feature. The MotionSqueeze module is inserted into ResNet and evaluated on Something-Something-V1, Something-Something-V2 [37], Kinetics [54], and HMDB51 datasets [40].

Kalfaoglu et al. [22] proposed a method which obtained highest accuracy on both HMDB51 [40] and UCF101 [39] datasets with 85.10% and 98.69%. The most important thing in this study is that the authors replace the conventional temporal global average pooling (TGAP) layer by the bidirectional encoder representations from transformers (BERT) layer. This replacement utilize the temporal information with BERT's attention mechanism. They declared that TGAP ignores the order of the temporal features, and BERT can focus on the important temporal features. The proposed network removed temporal global average pooling at the end of the proposed 3D CNN architecture. A learned positional encoding was added to the extracted features to maintain the positional information. The two last parts of the architecture is multihead attention a classification. Then, they also proposed some features reduction blocks. Attention is a useful tool in many fields of computer vision. A novel W3 (what-where-when) video attention module [55] including a channel-temporal attention *M*^*c*^ and a spatiotemporal attention *M*^*s*^ was proposed for the action recognition problem. An average-pooling and a max-pooling are used to aggregate global spatial information. The output is fed into a shared MLP network to exploit the interchannel relationship. To model the temporal dynamics of objects, a channel temporal attention with two layers of 1D convolutions is computed. With spatiotemporal attention, an average-pooling and max-pooling are used as in channel-temporal attention to exploit spatial feature maps. The features are concatenated and fed into a 2D convolution to obtain frame-level spatial attention. To obtain the temporal attention, two 3D convolutional layers is applied with the frame spatial attention of previous step. The W3 attention module was integrated the ResNet50-based TSM [14].

The backbone CNN network plays a vital role in many recent action recognition systems. Martinez et al. [56] changes the last layers of the backbone network to improve the representation capacity. The important information is maintained in global feature branch. The global feature branch consists a global average pooling and a linear classifier. The average pooling aggregates the spatial and temporal information of the video. In the discriminative filter bank, the filters are includes 1 × 1 or ×1 × 1 × 1 convolutions and global max pooling to compute the highest activation value. The third branch is local detail preserving feature branch. A bilinear upsampling operation are applied to double the resolution of the features. A skip connection is add from the features of stage 4. Two backbone networks (2D TSN [57] and inflated 3D [38]) were used to evaluate the proposed module with Something-Something-V1 [58] and Kinetics-400 [38]. The temporal modeling methods based on 3D CNN requires a large number of parameters and computations. Lee et al. [59] proposed VoV3D which is an 3D network with an effective temporal modeling module for temporal modeling. The module names temporal one-shot aggregation (T-OSA). The T-OSA use many 3D convolutions with different receptive fields. All the output features are concatenated and reduced dimension by a 1 × 1 × 1 convolution. In addition, the authors proposed a depthwise spatial-temporal module which decomposes a 3D depthwise convolution into a spatial depthwise convolution and a temporal depthwise convolution for making a more lightweight and efficient network. Something-Something-V1, Something-Something-V2 [58], and Kinetics-400 [38] was used to evaluate.

Zhao and Snoek [60] proposed a single two-in-one stream network to reduce the complex computation of two stream network. The network processes both RGB and optical flow in a single stream. The most important contribution in this work is motion condition layer and motion modulation layer. The motion condition layer maps flow inputs to motion condition Ψ. Then, the motion condition Ψ is fed into the motion modulation to learn two affine transformation parameters (*β*, *γ*). These parameters are used to influence the appearance network as below formula ℳ^2^(*F*^*rgb*^)=*β*⊙*F*^*rgb*^+*γ*, where *F*^*rgb*^ is the RGB feature maps and ⊙ is an element-wise multiplication operation. Instead of using deeply stacking convolution layers, Huang and Bors [61] proposed region-based nonlocal (RNL) to exploit long-range dependencies. The RNL operation is used to compute the relation between two positions based on their features and the neighboring features. The feature of each position is computed from all neighboring positions. The RNL operator is embed into a residual block as *z*=*yW*_*z*_+*x*. In addition, the RNL block is combined with SE [62] block to exploit spatiotemporal attention and channel attention. Two backbone networks are used to implement the proposed RNL, including ResNet-50 [52] and temporal shift modules (TSM) [14]. The network was evaluated on Something-Something-V1 [37] and Kinetics-400 [38]. Furthermore, OmniSource [63] trains video recognition model using web data, such as images, short videos, and long videos. The methods train a 2D teacher network and a 3D teacher network to filter the the web data that have lo confidence scores. Hua et al. proposed a dilated silhouette convolutional network (SCN) [64] for human action recognition in video. The silhouette boundary curves of the moving subject are extracted, and then, the silhouette curves are stacked as a 3D curve volume. The curve volume is resampled to a 3D point cloud to represent the spatial and temporal information of actions.

### 2.4. Methods Based on 3D Multistream Network

Multistream networks can exploit different types of features in human action recognition. Spatiotemporal and motion information are two important features of human action recognition. A two-branch network has two branches, including the RGB branch and flow branch. The RGB branch exploits the visual structure of scenes and objects, while the flow branch exploits the motion of objects. Many recent proposed methods use a 3D CNN to exploit spatiotemporal information and a flow stream to exploit motion information [24, 26, 38]. The two-stream network obtains state-of-the-art accuracy by using RGB and flow images as input. However, each stream is usually trained individually and the optical flow requires a heavy computation. Therefore, some approaches try to construct a two-stream network more efficiently [23, 65].  Figure 3 shows a two-stream network architecture that are used in many recent approaches.

To pay different types of attention, a two-stream attention [26] was proposed using the visual attention mechanism. The network contains two streams. The first stream is the temporal feature stream which inputs an optical flow image sequence. An LSTM and a temporal attention are used to aggregate the information of the optical flow image. The second stream is a spatial-temporal feature stream. This stream uses an LSTM architecture to encode the temporal relationship. The spatial features are extracted by some convolutions. Then, the spatial attention assigns an important location for the next step of feature generation and the temporal attention is used to focus the temporal frames. The method was evaluated on UCF11 [66], UCF Sports [67], and jHMDB [68]. An approach convert 2D classification networks into 3D ConvNets. The network is named as Two-Stream Inflated 3D ConvNets (I3D) [38]. They inflated all the filers and pooling kernels of the 2D architecture by enlarging a temporal dimension. To pretrain the 3D model on the ImageNet dataset, the authors converted an image into a video by copying it many times. The network has two streams. The first stream uses RGB inputs and the second one use flow inputs. The two networks are trained separately and the results are averaged. A two-pathway convolutional neural network [24] was proposed by Huang et al., namely Fine and Coarse. In the fine branch, motion information of raw input is extracted by a motion band-pass module. The extracted motion is fed into a backbone CNN [69] to learn the fine-grained motion features. On the other hand, the coarse branch is used to learn coarse-grained information. The raw frames are downsampled and fed into a backbone CNN to exploit coarse-grained features. In order to merge the features from two branches, a lateral connection module was established. The proposed method was evaluated on Something-Something-V1 [37], Kinetics-400 [38], UCF101 [39], and HMDB51 dataset [40]. A combination of RGB, flow, pose, and pairwise stream [70] was proposed to improve the performance of the action recognition system. The network includes two branches. The first branch uses CD3 [71] and I3D [38] as backbone networks to extract spatial and temporal information. In the second branch, a pairwise stream learns the spatial relationship between the subject who perform the action and the surrounding objects. In addition, a pose stream inputs keypoint images. Keypoint images provide the connected key body parts of a person. The predicted results are obtained by using the late fusion method. The network was evaluated on UCF101 [39] and HMDB51 datasets [40].

Optical flow requires high computing. A proposed approach [23] mimics the motion stream using a standard 3D CNN. They introduced two learning strategies, namely Motion Emulating RGB Stream (MERS) and Motion-Augmented RGB Stream (MARS). In the first strategy, a flow network is trained to classify actions using optical flow clips. Then the MERS is trained to mimic the flow stream using only RGB frames. The last layer of MERS is trained by using the imitative flow features. In the second strategy, a flow stream (teacher) uses optical flow clips to train. Next, the teacher network is frozen its weight and MARS (student) is trained with RGB frames as input. Since only RGB frames are used as input in the testing phase, the network avoids the high computation of optical flow. The optical flow requires a high computation cost. Stroud et al. [65] introduced Distilled 3D Network (D3D) which obtained high performance without optical flow computation during inference. The D3D combines motion information in the temporal stream into the spatial stream. This leads the spatial to behave like the temporal stream. D3D trains two networks, including a teacher network and a student network. The teacher network is a learned temporal stream of a two-stream network and the student network is a spatial stream. The knowledge of the teacher network is distilled into the student network during the training phase.

One of the problems of a two-stream network is to exploit the complementary information between two streams [25]. To solve this issue, Zhang et al. proposed a cross-stream network [25]. Two similar backbone networks are used to extract structure and motion features. Then, a cross-stream connection block is used to compute the correlation between the appearance and motion features. The classification scores are obtained by a classifier which inputs the extracted features of previous blocks. The cross-stream network is evaluated on UCF101 [39] and HMDB51 datasets [40] and Something-Something-V2 [58]. The most popular multimodality method fused its stream at the last stage of the model. A cross-modality [72] exchanges information between modalities in a more effective way. The proposed network has two branches. Instead of averaging the scores of the two branches, several cross modality attention (CMA) blocks are added after some stage of the network. The CMA matches a query of the first modality with key-value pairs of the second modality.

A very deep network [73] uses residual learning to encode spatial-temporal information human action recognition videos. The network, residual spatial-temporal attention network (R-STAN), includes two streams. Since the computation of optical flow has high cost, RGB Difference images are used to extract motion information. The RGB Difference images are computed by applying a element-wise subtraction operation between two frames. The network is constructed of many residual spatial-temporal attention blocks, including a residual block and a temporal and a spatial attention module. A feature map is processed as *M*′(*x*)=*M*⊙*A*_*T*_⊙*A*_*S*_, where *M* and *M*′ are the input and output feature maps and *A*_*T*_ and *A*_*S*_ are the temporal and spatial attention, respectively. Two standard datasets (UCF101 [39] and HMDB51 [40]) was used to evaluate the proposed method. A proposed neural network [74] computed the local and global representations parallel. Therefore, the feature maps are processed in local path and global path. In the first path, the local features *x*_*l*_ are updated from *x*_*l*−1_ and global vector *g*_*l*−1_. In the second one, the global vector is updated with local feature *x*_*l*_. Next, they proposed a local and global combination classifier to make the final prediction by combining the local and global representations. Finally, they proposed two different local and global diffusion networks, namely LGD-2D and LGD-3D. The difference between the LGD-2D and LGD-3D is that the input of the first one is *T* noncontinuous frames while the input of the second is *T* consecutive frames. In addition, LGD-2D and LGD-3D use 2D convolution and 3D convolution, respectively. They evaluated on two datasets, namely Kinetics-400 [38] and Kinetics-600 [75]. They also experienced on two of the most popular video action recognition datasets UCF101 [39] and HMDB51 [40].

Instead of training different networks separately, Zhou et al. [76] constructed a probability space from which a spatial-temporal fusion strategy can be derived. The authors introduced spatial-temporal fusion strategies that obtained high performance on poplar datasets. To exploit the mutual correlations in the video, an attention mechanism [77] is used in the 3D convolutional network. The authors proposed a temporal and spatial attention submodule and then used these attentions to construct the temporal and spatial deformable 3D convolutional network. Both 3D convolutional networks can learn temporal and spatial information as well as static appearance. A proposed model [78] used pose information to predict actions. First, they used the PoseNet approach with ResNet backbone to obtain estimated pose keypoints for each human in a frame. The backbone network used is ResNet50 with a 3D version. They added a feature gating module and did not apply temporal downsampling in any layer of the backbone network to improve the performance. The authors tried to avoid training three models separately since the input included RGB, flow, and pose data. They proposed a multiteacher framework in which its input can be RGB, flow, or pose. They evaluated on three benchmark datasets, including Kinetics-600 [38], UCF101 [39], and HMDB51 [40],

### 2.5. Convolution-Free Approaches

The 2D network is very successful in capturing the spatial features. However, the motion information is still missed. 3D convolution network is used to encode spatial-temporal information in videos but it requires a high computation cost. Transformer was proposed for natural language processing and then adopted for computer vision. It does not require heavily stacked convolutions to encode information, such as in [27–30].

A convolution-free model [27] that requires a smaller number of frames for inference. The model is based on a self-attention mechanism for capturing both spatial and temporal information. The authors separate the spatial attention and the temporal attention to reduce the computation and exploit temporal information better. Each input frame (*H* × *W*) of the network is split into nonoverlapping patches *N*=*HW*/*P*^2^, where the size of each path is *P* × *P*. Then, each patch representation is converted to query, key, and value vectors. To avoid expensive computation, spatial attention is applied between patches of the same image. The output representations of the spatial attention are applied to temporal attention. The proposed method was evaluated on Kinetics-400 [38]. They also reported the result on UCF101 [39].

To solve the heavy memory usage of the vanilla video transformer, a video transformer [28] was introduced to reduce the memory cost. The issue is solved by applying a spatial and temporal multihead separable-attention (MSA) sequentially *MSA*(*S*)=*MSA*_*s*_(*MSA*_*t*_(*S*)). Moreover, the authors solved the redundant information problem of the temporal dimension. Instead of using temporal average pooling or 1D convolutions with stride 2, they proposed a topK pooling which selects topK based highest standard deviation. They evaluated on 6 different datasets (Kinetics-400 [38], Kinetics-700 [79], Something-Something-V2 dataset [37], Charades [80], UCF101 [39], and HMDB51 [40]).

A convolution-free model is faster than 3D convolutional networks, namely, TimeSformer [30]. Each input frame is split into *N* nonoverlapping patches same as in [27]. The spatiotemporal position of each patch is encoded by a learnable positional embedding *e*_(*s*)_^*pos*^ ∈ *ℝ*^*D*^. Each patch *X*_*p*,*t*_ is mapped into an embedding vector *z*_(*p*, *t*)_^(0)^. The TimeSformer has *L* blocks and a set of query, key, and value vectors is computed from **z**_(*p*, *t*)_^(*l* − 1)^ for each block. In this study, the authors proposed a more efficient spatiotemporal attention. A temporal attention is applied, then, the output is fed into a spatial attention. The TimeSformer was evaluated on Kinetics-400 [38], Kinetics-600 [81], Something-Something-V2 datasets [37], and Diving48 [82].

Akbari et al. [29] introduced a convolution-free Transformer architecture, namely Video-Audio-Text Transformer (VATT). The input video clip is split into a sequence of ⌈*T*/*t*⌉·⌈*H*/*t*⌉ · ⌈*W*/*t*⌉ patches. The position of each location (*i*, *j*, *k*) is encoded as *e*_*i*,*j*,*k*_=*e*_Temporal_i__+*e*_Horizontal_*j*__+*V*_ertical_*k*__, and Multi-Head-Attention applies the self attention on the input. Multilayer perceptron includes two dense linear projections with a GeLU activation. The common space projection contains a linear projection, and a two-layer projection with ReLU activation functions in between. The proposed method was evaluated on UCF101 [39], HMDB51 [40], Kinetics-400 [38], Kinetics-600 [75], and Moments in Time [83].

## 3. A Comparison of Methods

First, we compare recent methods on two benchmark datasets, including UCF101 [39] and HMDB51 [40]. These are the two most popular human action datasets that have been used to evaluate the performance of the proposed methods as shown in Table 2. We group the proposed methods by year. In 2019, the local and global diffusion network achieved the best result with 98.20% and 80.50% on UCF101 and HMDB51, respectively. Their network tried to learn local and global feature in parallel, and these features are diffused effectively. In 2020, Kalfaoglu et al. [22] obtained impressive results with 98.69% and 85.10% on UCF101 and HMDB51, respectively. The replacement of the conventional temporal global average pooling layer with the bidirectional encoder representations from the Transformers layer increase the performance of 3D convolutional neural networks. In 2021, a three-stream network obtained 99.00% on the UCF101 dataset. In this year, many approaches introduced a new model for human action recognition with a convolution-free architecture, such as VATT [29], VidTr [28], STAM [27], and TimeSformer [30].

Table 3 compares recent approaches on Something-Something-V1 and Something-Something-V2. TSM [84] is one of the most effective methods which obtains both high efficiency and high performance because it obtains the performance of a 3D network with the complexity of a 2D network. TSM uses a simple temporal shift module to exploit a temporal relationship with zero extra computation and zero extra parameters. It obtains 52.60% and 66.00% top-1 accuracy on Something-Something-V1 and Something-Something-V2, respectively. Another method TDN [51] obtained state of the art on the Something-Something-V1 and Something-Something-V2 with 56.80% and 68.20%. TDN focus on capturing local and global motion for action recognition.

## 4. Benchmark Datasets

Benchmark datasets play a vital role in estimating the performance of proposed methods. The scope of the problem as well as a fairly comparison are provided by the dataset. For human action recognition, there is a wide range of benchmark datasets in common use. We briefly review the most well-known datasets and their information (size, average duration, action classes, and resolution) for human action recognition. These datasets are grouped into three categories such as simple, clip-level, and video-level.  Table 4 provides a summary of these datasets.

### 4.1. Simple Datasets

The two popular datasets which are most used with traditional methods are KTH [1] and Weizmann [2]. However, these datasets obtained absolute accuracy [102, 103] because the background is static and simple and one person performs an action in each video. Then, some more realistic datasets were proposed such as Hollywood [90] and Hollywood2 [91].

KTH [1] is a video dataset including 2391 videos. The dataset was performed by 25 different people in four different scenarios. The whole dataset (https://www.csc.kth.se/cvap/actions/) includes six human actions: walk, jog, run, box, hand-wave, and hand clap.

Weizmann [2] is a video dataset which was performed with nine people. Each participant performs 10 actions such as run, walk, jump, skip, jack, jump-forward, jump-in-place, side, wave-two-hand, and wave-one-hand. This dataset (http://www.wisdom.weizmann.ac.il/%20vision/SpaceTimeActions.html) includes 90 videos.

Hollywood [90] is a human action dataset taken from 32 movies. This dataset (https://www.di.ens.fr/%20laptev/download.html) has eight action classes with 233 training video samples and 211 testing video samples.

Hollywood2 [91] is a human action dataset with 3669 video clips. This dataset (https://www.di.ens.fr/%20laptev/actions/hollywood2/) includes 12 classes of actions and 10 classes of scenes with approximately 20.1 hours of video which is taken from 69 different movies.

### 4.2. Clip-Level Datasets

The number of actions of previous datasets is small, and the actions are simple. Therefore, some datasets such as UCF101 [39], HMDB51 [40], and J-HMDB [68] were introduced to provide a higher variety of actions. However, the samples are short clips, and a single action is captured. Then, some large-scale datasets, such as Charades [80], Something-Something [37], Kinetics [54], Kinetics-600 [75], Kinetics-700 [79], Diving48 [82], Moments in time [83], HACS [93], HVU [48], and AViD [94], have been introduced. These datasets allow to train a deep convolutional neural network from scratch.

UCF101 [39] has 101 action classes and has split into five categories: human-object interaction, body-motion only, human-human Interaction, playing musical instruments, and sports. It includes 13320 clips and 1600 minutes of video data. All videos (https://www.crcv.ucf.edu/data/UCF101.php) are downloaded from YouTube and have a fixed resolution of 320 × 240.

HMDB51 [40] has 51 action categories with 6,766 video clips (https://serre-lab.clps.brown.edu/resource/hmdb-a-large-human-motion-database/) which are extracted from different sources. There are five types of action, including general facial actions, facial actions with object manipulation, general body movements, body movements with object interaction, and body movements for human interaction. The height of all the frames is 240 pixels. To maintain the original aspect ratio of the video, the width was scaled accordingly to the height.

J-HMDB [68] is extracted from the HMD51 dataset [40]. Not only a dataset for human action recognition but also the J-HMDB is provided for pose estimation and human detection. The dataset (http://jhmdb.is.tue.mpg.de/) contains 21 classes with 31,838 annotated frames. Each action has 36–55 video clips, and each clip includes 15–40 frames.

MPII Cooking [92] is a dataset of cooking activities. The dataset (https://www.mpi-inf.mpg.de/departments/computer-vision-and-machine-learning/research/human-activity-recognition/mpii-cooking-2-dataset) contains 65 different cooking activities which are performed by 12 participants. In total, the dataset has 44 videos with 9 hours in length.

Charades [80] is a dataset of casual everyday activities of 267 people in their homes. The dataset has 9,848 videos with an average length of 30 seconds. It includes 157 action classes and is split into 7,985 videos for training and 1,863 videos for testing (https://prior.allenai.org/projects/charades).

Something-Something [37] includes 108,499 videos (https://20bn.com/datasets/something-something/v1) in V1 and 220,847 videos (https://20bn.com/datasets/something-something) in V2. Both versions have 170 action classes. The duration of a video is from 2 to 6 seconds. The dataset is divided into three parts, including training, validation, and testing set.

Kinetics [54] (Kinetics-400 [38]) has 400 human action classes, and each class has at least 400 video clips. All clips were taken from YouTube. The actions in the dataset are the human-object interactions or human-human interactions. The dataset (https://deepmind.com/research/open-source/kinetics) has 306,245 videos and is split into three parts for training, validation, and testing.

Kinetics-600 [75] is a large-scale, high-quality dataset. The dataset (https://deepmind.com/research/open-source/kinetics) was taken from YouTube with 500K video clips. It has 600 human action classes with at least 600 video clips for each class. The length of each clip is about 10 seconds.

Diving48 [82] has 48 classes of 48 different diving actions. The dataset (http://www.svcl.ucsd.edu/projects/resound/dataset.html) has 18,404 video clips which contain 16,067 clips for training and 2,337 clips for testing. All clips were taken without background objects and the scenes contain a board, a pool, and a spectator in the background.

Kinetics-700 [79] is an extension of the human action dataset Kinetics-600 [75]. The extended dataset (https://deepmind.com/research/open-source/kinetics) has 700 classes and was taken from YouTube. Each class of dataset has at least 600 video clips which have a variable resolution as well as frame rate.

Moments in time [83] is a human-annotated dataset with 339 different classes. This is a large-scale dataset with one million videos, and each video corresponds with an event occurring in three seconds. The dataset (http://moments.csail.mit.edu/) is split into 802,264, 33,900 and 67,800 videos for training, validation, and testing, respectively.

HACS [93] is a large-scale dataset for human action recognition. It contains 1.5M clips which are sampled from 504K untrimmed videos. All clips (http://hacs.csail.mit.edu/) in this dataset have a two-second duration with 200 action categories.

HVU [48] is a multilabel and multitask video dataset which aims to describe the whole content of a video. The dataset includes approximately 572K videos with real-world scenarios. This dataset (https://holistic-video-understanding.github.io/) is split into 481K videos for training, 31K for validation, and 65M for testing.

AViD [94] is a video dataset for human action recognition. The main difference of this dataset is that it is collected from many different countries. This dataset (https://github.com/piergiaj/AViD) contains 410K training clips and 40K test clips. The duration of each clip is from 3 to 15 seconds.

### 4.3. Video-Level Datasets

With the development of deep models, some large-scale datasets were introduced such as Sport1M [95]. However, this dataset only focuses on Sports actions. Recently, other action datasets have been introduced with larger samples and temporal duration such as ActivityNet [96], AVA [100], AVA-Kinetics [101], DALY [97], EPIC-Kitchens [99], MPII Cooking [92], and YouTube-8M [98].

Sport1M [95] includes 1 million YouTube videos. The dataset (https://cs.stanford.edu/people/karpathy/deepvideo/) contains 487 classes of sports. There are 1000–3000 videos in each class.

ActivityNet [96] is a benchmark dataset for human activity understanding. The dataset (http://activity-net.org/index.html) contains human activities in their daily living. With 849 video hours, ActivityNet provides 200 activity classes. Each class has an average of 137 untrimmed videos. Most of the videos have a duration between 5 and 10 minutes and a half of the video has a resolution of 1280 × 720.

DALY [97] is a dataset for action localization in space and time. The dataset (http://thoth.inrialpes.fr/daly/) lasts about 31 hours of YouTube videos with 10 everyday human actions.

YouTube-8M [98] is a multilabel video classification dataset. The dataset (http://research.google.com/youtube8m/) includes 8,264,650 videos. With 500,000 hours of video, YouTube-8M contains over 1.9 billion video frames and 4,800 classes.

EPIC-Kitchens [99] was recorded by 32 participants in their kitchens. The participants comes from 10 different countries. The dataset (https://epic-kitchens.github.io/2020-55.html) has 55 hours of videos which include 11.5M frames. The videos have a resolution of 1920 × 1080; however, there are 1% of the dataset was recorded at 1280 × 720 and 0.5% at 1920 × 1440.

AVA [100] is a video dataset in which theactions are assigned in space and time. In addition, each person in the video is annotated with multiple labels. This dataset (https://research.google.com/ava/) contains 437 different videos of realistic scenes and action complexities. Each video is taken from the 15th to 30th minute time and has 900 frames. It is divided into 239 videos for training, 64 videos for validation, and 134 videos for testing, roughly a 55 : 15 : 30 split.

AVA-Kinetics [101] is an extension of the AVA dataset [100] with new videos from the Kinetics-700 [79] annotated with the AVA action classes. The AVA-Kinetics (https://research.google.com/ava/) has 238,906 videos which is split into 142,475 videos for training, 32,529 videos for validation, and 64,902 videos for testing.

## 5. Open Research Problems

In the previous sections, we discuss the recent proposed methods and benchmark datasets for human action recognition with RGB data video. In this section, we will introduce some of the potential research problems in this field.

 
*Data for human action recognition* RGB videos are widely used in most methods for action recognition because these data are very popular and acquired with a low cost. However, other types of data provide more information for action recognition, such as skeleton, depth, infrared sequence, and point cloud. Skeleton data provide the trajectories of human body joints. Depth and point cloud data capture 3D structure and distance information. Infrared data provide data in a dark environment. Therefore, we cannot exploit color or texture in infrared data.
 
*Pose estimation* detects the location of human body joints in images. The skeleton data provide the body structure and pose of the object; therefore, we have more information for human action recognition. The skeleton data are obtained by using pose estimation on RGB videos or depth data.
 
*Combination* of different data types, such as RGB data with depth data or skeleton data with depth data, provides rich information for learning models. The RGB video data provide spatiotemporal features while depth data provide the 3D structure and depth information. We also combine different features of different models to get better performance.

## 6. Conclusions

In this survey, we provided a review of recent deep learning-based methods for human action recognition with RGB video data. We categorized recent approaches into five different groups, including 2D CNN-based methods, RNN-based methods, 3D single-stream network-based methods, 3D multistream network-based methods and convolution-free-based methods. More recently, a pure vision transformer with a convolution-free network has shown to be effective for human action recognition and various fields of computer vision. Therefore, we discussed recent transformer-based methods. We compared the accuracy of recent methods on four popular datasets, including UCF101, HDMB51, Something-Something-V1, and Something-Something-V2. We also discussed a wide range of benchmark datasets for human action recognition that are used in recently proposed methods. Lastly, we provide some potential research directions for human action recognition.

## Figures and Tables

**Figure 1:** The structure of the survey.

**Figure 2:** 3D single-stream network.

**Figure 3:** 3D two-stream network.

**Table 1:** Summary of the related survey articles.

Survey	Year	Scope							Contributions
		Handcrafted	2D CNN	RNN	3D single-stream	3D multistream	Convolution-free	Datasets	
[5]	2010	✓						✓	(i) We categorise five aspects of deep learning methods for human action recognition (ii) Convolution-free approaches are first reviewed in our work (iii) A detailed review of popular benchmark datasets for action recognition
[6]	2019	✓	✓	✓	✓	✓		✓	
[7]	2019							✓	
[8]	2019	✓	✓	✓				✓	
[9]	2020		✓	✓	✓	✓		✓	
[10]	2020							✓	
[11]	2020	✓						✓	
[12]	2021							✓	
[13]	2021	✓	✓	✓				✓	
Our	2021		✓	✓	✓	✓	✓	✓	

**Table 2:** Accuracy of different methods on UCF101 and HMDB datasets.

Method	Year	Method	UCF101	HMDB
Carreira and Zisserman [38]	2017	Two-stream I3D	98.00	80.90
Zhou et al. [47]	2018	Mixed 3D CNNs, 2D CNNs	94.70	70.50
Zhang et al. [43]	2019	SoSR + ToSR (TSN [84], ResNet [52])	92.13	68.30
Ge et al. [44]	2019	Attention + ConvLSTM	92.39	66.37
Pan et al. [17]	2019	TR-LSTM (Inception-V3 [85])	93.80	63.80
Liu et al. [73]	2019	R-STAN(ResNet101 [52], temporal and spatial attention)	94.50	68.70
Wang et al. [50]	2019	I3D, LSTM	95.10	—
Lin et al. [14]	2019	TSM (TSN [84])	95.90	73.50
Jiang et al. [31]	2019	STM (CSTM, CMM, TSN [84], ResNet50 [52])	96.20	72.20
Chi et al. [72]	2019	CMA (attention)	96.50	—
Zhang et al. [25]	2019	CSN (TSN [84])	97.40	**81.90**
Hong et al. [70]	2019	I3D [38]/CD3 [71] (RGB, flow, pairwise and pose)	98.02	80.92
Crasto et al. [23]	2019	MARS + RGB + Flow	98.10	80.90
Qiu et al. [74]	2019	LGD-3D two-stream	**98.20**	80.50
Piergiovanni and Ryoo [34]	2019	Fully-differentiable convolutional layer	—	81.10
Kwon et al. [53]	2020	MSNet (ResNet50 [52])	—	77.40
Liu et al. [45]	2020	STS + attention LSTM	92.70	64.40
Majd and Safabakhsh [19]	2020	*C* ^2^ *LSTM*	92.80	61.30
Huang and Bors [21]	2020	TSN (squeeze and excitation operation)	95.20	71.50
Li et al. [77]	2020	Attention (ResNeXt-101 [86])	95.90	72.20
Zhou et al. [76]	2020	Probability space	96.50	—
Zhu et al. [49]	2020	FAST-GRU	96.90	75.70
Diba et al. [48]	2020	HATNet (2D ResNet50, 3D ResNet18)	97.80	76.50
Zhang et al. [33]	2020	PANet (ResNet101 [52], TSM [14])	97.20	77.30
Duan et al. [63]	2020	2D network (ResNet50 [52]), 3D network (SlowOnly [87])	97.52	79.02
Stroud et al. [65]	2020	D3D (S3D-G [88])	97.60	80.50
Li et al. [32]	2020	CIDC (ResNet50 [52])	97.90	75.20
Li et al. [78]	2020	PoseNet, ResNet50 (3D), multiteacher network	98.20	82.00
Gowda et al. [36]	2020	MobileNet, MLP, LSTM	98.60	84.30
Kalfaoglu et al. [22]	2020	BERT, 3D convolution architecture	**98.69**	**85.10**
Akbari et al. [29]	2021	VATT	89.60	65.20
Xu et al. [35]	2021	MotionNet [41] + OFF [42]	91.50	67.90
Li et al. [28]	2021	VidTr (MSA, topK-based pooling)	96.70	74.40
Sharir et al. [27]	2021	STAM (spatial and temporal attention)	97.00	—
He et al. [18]	2021	DB-LSTM (ID3 [38])	97.30	81.20
Huang and Bors [24]	2021	FineCoarse (TSM R50 [69])	97.60	77.60
Hua et al. [64]	2021	SCN (Mask R-CNN [89])	98.30	**85.10**
Sheth [46]	2021	Three-stream network + LSTM/Attention	**99.00**	—

Bold represents the best performance.

**Table 3:** Accuracy of different methods on Something-Something-V1 and Something-Something-V2 datasets.

Method	Year	Method	Something-V1		Something-V2	
			Top-1	Top-5	Top-1	Top-5
Zhou et al. [15]	2018	TRN (2-stream TRN)	42.01	—	55.52	83.06
Jiang et al. [31]	2019	STM (CSTM, CMM, TSN [84], ResNet50 [52])	50.70	80.40	64.20	89.80
Lin et al. [14]	2019	TSM (TSN [84], ResNet50 [52])	52.60	81.90	66.00	90.50
Tran et al. [20]	2019	CSN (ResNet3D [52])	53.30	—	—	—
Martinez et al. [56]	2019	2D TSN [57], inflated 3D [38]	**53.40**	81.80	—	
Li et al. [32]	2020	CIDC (ResNet50 [52])	—	—	56.30	83.70
Zhou et al. [76]	2020	Probability space	—	—	62.90	88.00
Perez-Rua et al. [55]	2020	W3 (ResNet50-TSM [14])	52.60	81.30	66.50	90.40
Lee et al. [59]	2020	VOV3D-L (T-OSA)	54.70	82.00	67.40	90.50
Kwon et al. [53]	2020	MSNet (ResNet50 [52])	55.10	84.00	67.10	91.00
Sudhakaran et al. [16]	2020	GSM (InceptionV3 [85])	55.16	—	—	—
Zhang et al. [33]	2020	PANet (ResNet101 [52], TSM [14])	55.30	82.80	66.50	90.60
Wang et al. [51]	2020	TDN (short- and long-term TDM)	**56.80**	84.10	**68.20**	91.60
Huang and Bors [61]	2021	RNL (ResNet50 [52], TSM [14])	54.10	82.20	—	—
Huang and Bors [24]	2021	FineCoarse network (ResNet [52])	**57.00**	83.70	—	—

Bold represents the best performance.

**Table 4:** Some benchmark datasets for human action recognition.

Dataset		Year	Samples	Mean length	Actions	Resolution
Simple	KTH [1]	2004	2391	4 sec	6	160 × 120
	Weizmann [2]	2005	90	Len	10	180 × 144
	Hollywood [90]	2008	430	Len	8	—
	Hollywood2 [91]	2009	3669	Len	12	—

Clip-level dataset	UCF101 [39]	2012	13,320	7.21 sec	101	320 × 240
	HMDB51 [40]	2013	6,766	—	51	—– × 240
	J-HMDB [68]	2013	31,838	1.4 sec	21	320 × 240
	MPII cooking [92]	2012	881,755	Len	65	1624 × 1224
	Charades [80]	2016	9,848	30 sec	157	671 × 857
	Something-Something-V1 [37]	2017	108,499	4.03 sec	174	—– × 100
	Something-Something-V2 [37]	2018	220,847	4.03 sec	174	—– × 240
	Kinetics-400 [38]	2017	306,245	10 sec	400	Variable resolution
	Kinetics-600 [75]	2018	495,547	10 sec	600	Variable resolution
	Kinetics-700 [79]	2019	650,317	10 sec	700	Variable resolution
	Diving48 [82]	2018	18,404	Len	48	—
	Moments in time [83]	2019	1,000,000	3 sec	339	340 × 256
	HACS [93]	2019	1.55M	2 sec	200	—
	HVU [48]	2020	572K	10 sec	739	—
	AViD [94]	2020	450K	3–15 sec	887	—

Video-level dataset	Sport1M [95]	2014	1,133,158	5 min 36 sec	487	—
	ActivityNet [96]	2015	28,108	(5–10) min	200	1280 × 720
	DALY [97]	2016	8133	3 min 45 sec	10	1290 × 790
	YouTube-8M [98]	2016	1.9B	226.6 sec	4,800	—
	EPIC-kitchens [99]	2018	11.5M	1.7 hrs	149	1920 × 1080
	AVA [100]	2018	392,426	15 min	60	451 × 808
	AVA-kinetics [101]	2020	624,430	—	60	—

## Data Availability

The datasets generated during and/or analysed during the current study are available from the corresponding author on reasonable request.
